The article "The Positioning of Mental Health Education in Social Work under the Healthy China Strategy" was published in 2022. Journal: J Environ Public Health.

# The Positioning of Mental Health Education in Social Work under the Healthy China Strategy

**DOI:** 10.1155/2022/4338011

**Published:** 2022-06-21

**Authors:** Xiao Wang, Manyi Gu

**Affiliations:** Southwest Medical University, School of Humanities and Management, Luzhou, Sichuan 646000, China

## Abstract

In recent years, the world mental health movement has developed rapidly, and people are paying more and more attention to mental health. China has clearly put forward the major task of comprehensively promoting the construction of a Healthy China and building a Healthy China by 2035. However, in contrast, the research on mental health in Western countries started earlier than in my country, and for a long period of time, my country has followed the research results of Western mental health ideas. Every different culture has its own unique psychological content. Due to factors such as values, habitual behavior, region, and cultural background, it is necessary to deeply explore the mental health thought resources in Chinese culture and study the mental health thought in Chinese culture. It provides new directions and ideas for our country's psychological counseling and treatment, as well as mental health education and ideological and political education. This article starts from the basic concept of mental health education and sorts out the current research status at home and abroad. By analyzing the main ideas of mental health education work in the context of Healthy China, it explores the positioning of mental health education in social work, and finally, on the basis of strengthening the combination of Chinese culture and mental health thinking, making full use of localized mental health thought and applying it to practice, and drawing inspiration for the study of mental health thought in Chinese culture.

## 1. Introduction

Health is the basis of human survival and development, and it is the basic premise for people to achieve happiness. The national health level is also an important part of the national comprehensive national strength and national competitiveness and is an important strategic factor affecting the country's social and economic development [1]. The Proposal of the Fifth Plenary Session of the 19th CPC Central Committee on the formulation of the 14th Five-Year Plan for National Economic and Social Development and the Two-O Five-Year Vision Plan (hereinafter referred to as the Proposal) clearly proposes the major tasks of comprehensively promoting the construction of a Healthy China and building a Healthy China by 2035. The Healthy China strategy is a major strategic project designed to improve people's livelihood and is also a requirement and important part of China's socialist modernization. The implementation of the Healthy China strategy requires the concept of “people's health” running through the national development plan, realizes cross-departmental and cross-field cooperation and exchanges, and continuously promotes the concept of Healthy China in the process of realizing coconstruction and sharing by all people [2]. Thus it can be seen that the Healthy China strategy is not only lofty but also has rich connotation and has strong research significance. This is a major strategic plan made by the CPC Central Committee with Comrade Xi Jinping at its core to review the overall situation and assess the situation. Comprehensively promoting Healthy China construction fully embodies the development of the people-centered thought, is the relationship global strategic task of socialist modernization construction, is the inherent requirement of guarantee people enjoy a happy life, is the important security of national public security, to open the comprehensive construction of modern socialist country new journey, promotes the development of the new era of health quality, and realizes that the great rejuvenation of the Chinese nation the Chinese dream has great historical significance and practical significance [2].

Mental health is of great significance for individuals to promote their health and develop a healthy lifestyle. We believe that mental health refers to a set of concept systems about disease prevention, maintaining health, and striving to achieve the best state of life, which is the firmly believed concept of healthy life [3]. It contains an individual's view on what health is, the importance of health, factors affecting individual health, and ways to improve health. Individuals with different mental health can lead to different health behaviors, lifestyles, and health conditions. Social development is getting faster and faster, the competition is becoming more and more fierce, and the threat of psychological problems to health has been far greater than physical diseases. Health is an inevitable requirement for promoting the all-round development of human beings, a basic condition for economic and social development, an important symbol of the prosperity of the nation and national prosperity, and the common pursuit of the broad masses of the people. Therefore, in the context of the health China strategy, it is particularly important to study the positioning and role of mental health education in the overall health China strategy. This article aims to start with the meaning, classification, and goal of mental health education, analyze the problems of mental health in the overall background of Healthy China, and propose the improvement and countermeasures of mental health education, in order to improve the role of mental health education [3].

## 2. Mental Health Education

### 2.1. Meaning of Mental Health Education

Mental health education, according to the law of people's psychological activities, takes various methods and measures, mobilizes all internal and external positive factors, maintains individual mental health, and cultivates good psychological quality to promote the overall quality of education [4]. Mental health education is a new education concept, a new education model, and a multidimensional and multilevel education system. We can make the following analysis of its rich connotation.

From the perspective of content, mental health education includes two parts: psychological quality training and mental health maintenance [5]. Psychological quality is a relatively stable psychological characteristics, attributes, or qualities produced and developed in the interaction between individuals and the objective outside world on an innate basis, which is mainly composed of the combination of intellectual and nonintellectual factors [4]. The psychological quality of individuals reflects the development level of their psychological function, which determines the effect of individual intellectual activities but also determines the difficulty and level of individual social adaptation. Psychological quality plays an important and unique role in the three basic human qualities (physical quality, psychological quality, and social and cultural quality). The fundamental purpose of cultivating psychological quality is to promote the comprehensive development of people's quality. Only the comprehensive development of quality can have the development of a sound personality [6].  Figure 1 gives the causes of psychological stress in college students, and it can be seen that the stress factors of mental health are diverse, as shown in Figure 1 [5].

The maintenance of mental health is mainly to make individuals form and maintain a normal psychological state so as to adapt to the society, normal growth, and development [6, 7]. Specifically, one is to help people form self-regulation ability and maintain a normal psychological state; two to help the bad psychological state of people to restore normal state; three is to help psychologically unhealthy people to restore healthy state [7]. These two aspects of mental health education reflect the different levels of people's normal growth and development. Psychological quality training is mainly to make people can succeed and become talented; mental health maintenance is mainly to enable people to grow and develop normally, can adapt to the society, and can grow into healthy adults throughout the whole life growth stage of the mental health education system, as shown in Figure 2.

### 2.2. Classification of Mental Health Education

According to the different nature of mental health education, mental health education can be mainly divided into two categories: one is developmental education and the other is remedial education [7, 8].

Developmental education mainly refers to the process of psychological counseling personnel on the basis of understanding the general laws of individual psychological development, giving certain education and counseling for the tasks faced by people at different stages so as to properly solve their psychological contradictions and give full play to their psychological potential, so as to promote the smooth development of their physical and mental health. This is a kind of routine, preventive, and improving education; the object of education is the normal development of the people [7, 9].

Remedial education refers to the process in which psychological education cannot play a role; psychological counseling personnel give direct guidance and help to the problems in study, life, and adaptation, to diagnose and correct the relevant psychological disorders or minor mental diseases. This is a kind of corrective education, and the object of education is the people with psychological problems of different degrees [10].

### 2.3. Objectives of Mental Health Education

In recent years, China has made great achievements in the theoretical research and practice of mental health education and accumulated rich experience, but there is a lack of systematic research on the target system, especially the target content. The goal of mental health education is the guidance and basic basis of carrying out mental health education, which is the prerequisite for the correct and effective implementation of mental health education and is also a key link of mental health education planning [11].

The goals of mental health education can be divided into different types. According to the abstraction of the goal, it can be divided into general goal or specific goal [10]. According to the level of goals, it can be divided into primary goals, intermediate goals, and advanced goals. The overall goal of mental health education should reflect the basic requirements of mental health education and meet the requirements of educational training goals. Therefore, the general goal of mental health education can be summarized as follows: through mental health education, improving people's psychological quality, developing people's potential, cultivating people's optimistic psychological quality, relieving psychological confusion, and promoting the sound development of people's personality. The general goal of people's mental health education can be determined according to the task or the main staged topic to be solved. From the perspective of the goal level, the primary goal is to prevent and treat mental illness, the intermediate goal is to improve psychological adjustment, and the final goal is to promote psychological development.

### 2.4. Status and Function of Mental Health Education

#### 2.4.1. Mental Health Education Plays an Essential Role in the Development of Modern Education

From the perspective of dynamic balance, some scholars have proposed that mental health is essentially a process, and it is the normal operation of the balancing mechanism of the automatic adjustment of the psychological system. Some scholars believe that mental health is a necessary part of a person's overall health and is a continuous mental state. In this state, individuals have a vitality of life, positive inner experience, and good social adaptation. To give full play to the physical and mental potential and positive social functions of individuals, modern education is transforming the traditional education mode of imparting knowledge into a scientific education mode; the test-oriented education mode is transformed into a quality education mode. The fundamental purpose of quality education is to comprehensively improve the quality of all students. Quality education is based on physical quality education and psychological quality education, and psychological quality is the basic component of social and cultural quality. Psychological education is not only narrow mental health education but also psychological quality education. Psychological education plays a dominant role in the harmonious development of personality. Intelligence in psychological quality is an important basis for learning knowledge, and it needs to be the inner driving force of human development. Personality and self-awareness affect people's learning style and cultural structure. Psychological quality is the basic component of social and cultural quality, as shown in Table 1.

#### 2.4.2. Mental Health Education Occupies a Dominant Position in the Harmonious Development of Personality

In the process of individual socialization, the harmonious development of personality constitutes the core component of the overall quality. The criteria of personality health include at least three aspects: good realistic perception, a good understanding of self, and a positive attitude towards life [12]. A person with a healthy personality can correctly understand the real environment, have appropriate behavior and emotional response, have a good interpersonal relationship, can be self-pleasing, have basic accurate self-expression cognition and no inferiority, and can adjust and control your emotions; able to face life with a positive attitude, dare to bear setbacks, dare to overcome difficulties, and have good behavior. Such students can effectively conduct learning activities. A healthy personality is a basis for forming a good moral character, which is closely related to the efficiency of intellectual activities and is beneficial to promoting the development of physical health and aesthetic education. It is involved in the process of individual socialization adapted to modern society. It is the main task of psychological education in colleges and universities to help students develop their personality harmoniously by means of psychological counseling and psychological counseling, and traditional education is just ignored in this important aspect [13].

#### 2.4.3. Mental Health Education Plays a Leading Role in Developing Human Potential

The development of human potential is based on two aspects of accumulation: one is the genetic quality of human life evolution: the other is the spiritual wealth of human social practice and the “inheritance” of spiritual wealth is the sacred mission of education [14]. Education enables future generations to stand on the shoulders of their predecessors as soon as possible and promote the better development of human society. Developing people's potential is one of the purposes of quality education, which requires the professional knowledge and methods of psychological education and cannot be simply included in ordinary teaching. Every student is a talent whose potential remains to be developed. The key is to let each student understand his own intellectual structure and the corresponding means of development through the means of psychological education. There is a basic contradiction between adaptation and development, and the imbalance of this contradictory relationship will inevitably lead to mental health [15]. Psychological education focuses on the development of students' potential so as to drive the overall progress of students [12].

## 3. Mental Health Education at Home and Abroad

Internationally, humankind is in a period of great development, reform, and adjustment, where countries are interconnected and interdependent, and the world has a common destiny. When it comes to “mental health,” it is a product from the West. As early as the end of the 19th century, the Western traditional culture, which advocated scientism and humanism, specially studied “psychology” as a science [16]. In contrast, the scientific research on mental health in China does lag far behind. However, Chinese culture has long contained rich mental health ideas. Chinese culture provides a lot of valuable exploration and thinking about people's inner life, and Chinese culture carries a kind of reflexive knowledge. Although it has no specific psychological part in it, it contains many mental health thoughts and special ways of cultivating morality, strongly permeates the psychological customs of Chinese society, and constructs the unique psychological lifestyle in the Chinese cultural background [14].

### 3.1. Foreign Mental Health Research

The theoretical research and practice related to health concepts and health strategies in Western countries all started earlier. In the past half a century, the research content has been extended from the connotation and value of health and health fairness to the value of a healthy lifestyle, and the focus of health national strategy has also undergone many adjustments and improvements. Psychology originated in the West and in itself is rooted in Western culture. Various schools and theories of Western psychology reflect Western values and Western cultural values and have a strong Western cultural color [17]. Western psychology tries to follow and imitate the relatively mature natural science and then with the hegemony of the American psychology is their psychological knowledge system; this research is universal and applicable and is found to be the only applicable psychological system beyond the local culture [18].

These research results and experience abroad have provided us with rich information. Under the background of the current market economy construction, the mental health of the Chinese people is particularly important. For foreign experience and conclusions, we must choose to absorb and learn from it, take its essence, and discard its dross. This requires us to explore the localization of mental health thought in China by reasonably using the successful experience of mental health model in Western countries [15].

### 3.2. Domestic Mental Health Education

Chinese psychologists have long realized the importance of localization. As early as 1920, sociologist Yang Kaidao pointed out that one of the major flaws in Chinese social sciences was the blind use of foreign materials while ignoring domestic materials. Mental health thought is subordinate to psychology and is a branch of psychology. Research on mental health thought is also an important part of psychology research content; with the development of psychological localization, many scholars also explore the localization of mental health thought; in the localization of mental health thought, most scholars have followed the perspective of Chinese culture and the mental health thoughts in Chinese culture and analysis and also obtained many results. Shen Xiaomei believed that “mental health education is the use of modern educational methods by educators to help people understand the world beautifully, master psychological knowledge, analyze the causes of psychological problems, and prevent the occurrence of psychological problems, so as to improve their ability to understand themselves and promote physical and mental health.” In terms of the process of healthy growth, Wu Qiang believed that strengthening mental health education is the need for the development of the Internet era and the need to solve the psychological problems of college students.

Chinese psychologists began to gradually realize the positive influence of mental health thought in Chinese culture on the development of modern psychological science and made efforts to promote the development of the localization of mental health thought [19]. By reading a large amount of literature, it can be concluded that there are two main tendencies of various scholars: one is to completely deny the Western mental health idea and abandon Western psychology; the second is that the theoretical framework of Western scientific psychology when based on traditional culture. This article states that the first tendency exaggerates the role of Chinese culture, while the second view takes the essence of Chinese culture and Western mental health thought and discards its dross, which is more in line with the requirements of cultural innovation, more scientific and more in line with the reality [16].

In general, the research on the localization of mental health thoughts in China has been developing. The main research includes the exploration and arrangement of mental health thoughts in Chinese culture and the research on the unique psychological behavior of Chinese people since the late 1980s [20]. Localization of mental health thought research as part of the localization of psychology, and psychology localization is still in its infancy, mainly manifested in “the goal, strategy, and means to achieve the goal is still not clear, there is no unified program of action, not beyond the plight of localization and globalization.” That is to say, the research work on the localization of mental health thought in China is still in the initial stage, but it is undeniable that the localization of mental health thought in China has been developing [17].

### 3.3. The Healthy China Strategy

As an important social cause and people's livelihood project in the new era, the construction of Healthy China must provide concept first and lead its development with correct ideas. According to the 19th report “for the people to provide a full cycle health services” and “prevention first” spirit, and the deepening of the law of health medicine development and health national strategy international experience, we put forward the three basic ideas of the construction of Healthy China—health concept, health concept, and the concept of prevention first. The 2030 phase targets of the Healthy China Initiative are shown in Figure 3.

#### 3.3.1. The Concept of the Right to Health

Health is the basic demand and necessary condition for individual survival and development, and it is also the most important value orientation of human society. A person's health condition will directly affect his income ability and living standard and then affect the realization of his social and economic rights. Therefore, the right to health is regarded by the natural law school as an innate and irresistible basic human right, which is the basic premise of maintaining a better life for citizens. The right to health, as a basic human right, has long been protected by law in history. The right to health means health equity; that is, everyone has an equal right to health, which requires the state to assume the responsibility and obligation to protect people's health rights and interests and health equity. The right to health imposes three levels: the government to protect the right to health from the civil right, the government, and the right to respect every citizen's right to health from the political right. Under the Healthy China grand strategy, the national planning of mental health education for residents at the social level is shown in Figure 4.

#### 3.3.2. Big Health Concept

The report to the 19th National Congress of the Communist Party of China and the Outline of the “Healthy China 2030” Plan both advocates that building a Healthy China should focus on improving people's health, accelerate the transformation of the development mode in the health field, and maintain and protect people's health in an all-round and whole-cycle way. This is essentially advocating a new health concept—big health. “Great health” is the expansion and sublimation of the concept of “health.” Different from the traditional understanding of “no disease of the body is healthy,” “great health” pursues comprehensive health, including body, spirit, psychology, physiology, society, environment, and other aspects. It is a global concept put forward according to the development of the times, social needs, and changes in disease spectrum [18]. It focuses on human birth, aging, illness, and death, pays attention to various risk factors affecting health, and advocates self-health management and health environment management so as to reduce disease risks and promote the improvement of people's health levels. From the perspective of the areas of Healthy China, the core connotation of big health is as follows: the whole life cycle health covering the whole population, that is, the whole process of “from negative one year to life,” including gestation (maternal), childhood, adulthood, old age, and hospice care; the comprehensive health covering the whole population, that is, physical health, mental health, social adaptation health, lifestyle health, and living environment health. Mental health education is an important part of the big health concept, as shown in Figure 5.

#### 3.3.3. Prevention First Concept

The report to the 19th National Congress of the CPC proposed “putting prevention first and combining prevention and control,” which is based on the deepening of the understanding of the development laws in the health field. “Prevention first” concept under the guidance of health maintenance focuses on preventing and reducing the occurrence of disease to reduce the cost of Healthy China construction and improve people's happiness and has positive effects, both health and economic effects. Healthy China construction should always adhere to the basic concept and must be implemented in all aspects of the construction of Healthy China. In the popularization of a healthy life, more attention should be paid to the prevention and health care effects of physical fitness, strengthen health education, and improve the health literacy of all the people; in optimizing health services, attention should be paid to the disease prevention and control of comprehensive chronic diseases and health management and promote the equalization of basic public health services [19].

## 4. Countermeasures and Suggestions for Mental Health Education

### 4.1. The Current Challenges of Social and Mental Health

In 2020, the COVID-19 outbreak and epidemic around the world. China made full use of its significant advantages of concentrating resources to accomplish great tasks, gathered all social forces to fight the epidemic, and introduced a series of strong policies and measures [20]. Zone spreading work mechanisms of the State Council have issued the notice of coronavirus pneumonia epidemic emergency psychological crisis intervention guidelines notice, the notice about setting up the outbreak psychological assistance hotline, and printing COVID-19 epidemic psychological counseling work plan notice, guidance around different periods, different groups of psychological counseling, and crisis intervention work. It can be seen that psychological work has been raised to an unprecedented height in response to the epidemic. According to the Chinese report on national mental health development, the pressure on national mental health is increasing rapidly, as shown in Figure 6.

The phased assessment of mental health education on China's social psychological service system construction is also a challenge to China's social governance capacity. Under the current epidemic, the Chinese people of all ethnic groups have worked together in times of trouble, fully demonstrating the Chinese nation: the patriotic feelings of integrating the country, the spirit of mutual assistance from all sides, and the indomitable character of perseverance. Moreover, at the same time, the public also shows negative emotions and cognitive and behavioral performance such as group panic, confidence crisis, and moral anomie.

#### 4.1.1. Panic: Anxiety and Conformity Behavior

Major epidemics lead to a social state of emergency. The uncertainty, low incidence, and unconventional and rapid response to emergencies can easily lead to individual response failure and some specific response modes. Group panic, which is one of the specific response methods, may be emotional, such as anxiety, fear, powerlessness, and behavior, and may be conformity, panic, at a loss. The mental health of different ages is not identical, as shown in Figure 7.

#### 4.1.2. Crisis of Confidence: Overload of Information and Lack of Trust

Modern society is in the era of information explosion. Home isolation does not mean information isolation but instead makes people spend more time updating epidemic-related information. Through the collection and investigation of relevant data, it is found that 27.7% of the public spend more than 2 hours on epidemic-related information every day, and 39.8% of them update information more than 5 times. However, is more information the better? A striking contrast is that in 2003, when the SARS outbreak broke out, a related survey found that the proportion of the public updating information more than 5 times a day was 17.6%. Mainly based on TV and newspapers, the current channels for people to obtain information are the Internet, traditional newspapers, and TV. Therefore, the self-assessment anxiety level (37.29 points) is much lower than the anxiety level of the respondents under the current epidemic (40.75 points). On the one hand, information overload leads to increased psychological pressure; on the other hand, the degree of trust in various types of information is not high, and this uncertainty further causes panic. According to the results of this survey, the public has an average level of trust in the information of 3.44 points. Among them, the trust in official news and reports is the highest, the trust in the forwarding of messages from relatives and friends is the lowest, and the large websites and social platforms are in the middle. The specific data are shown in Table 2.

#### 4.1.3. Moral Anomie: Egoism and Social Indifference

Disaster will magnify the goodness of society, and it will also amplify the gray of a society. Since the outbreak of the epidemic, it can be seen that the people of the country donated money to the epidemic area, some businessmen embezzled, misappropriated, and delayed some officials to avoid others, and some patients deliberately concealed their trips, resulting in a large number of medical workers are infected. Under the “national system,” on the one hand, the concept of one province package one city “united city” is found in some areas. Talk about Hubei color change and even disclose the privacy information of returnees without authorization. These social phenomena have exposed some bad social mentalities to varying degrees.

### 4.2. Countermeasures and Suggestions to Strengthen Mental Health Education

#### 4.2.1. Improve the Social Service System

Clarify the basic public service orientation of social psychological services, implement the main body responsible for the construction of the social psychological service system, strengthen and improve the top-level design, formulate evaluation indicators, professional norms, and ethical codes for system construction, and coordinate the promotion of system construction. Strengthen the use of big data and cloud computing, and establish a social psychological service steward system. It is necessary to further explore the relevant social psychological indicators included in the government's basic services and scientifically measure the amount of financial support. This can start with some existing measurement indicators and select and supplement relevant indicators. It is suggested that the National Patriotic Health Campaign Committee should add relevant indicators of social psychological services and take the lead in introducing the relevant indicator system in the evaluation process of healthy cities so as to promote the improvement of the level of urban social psychological services. Of course, in townships and rural areas, different types of measurement index systems may need to be adopted, which requires further research.

#### 4.2.2. Increase Localization Research in Related Disciplines

Vigorously develop related discipline groups represented by health psychology, social psychology, and cultural psychology with Chinese characteristics, and cultivate scientific research and practical talents related to social psychological services. In particular, the research, practice, and talent training of community psychology, policy psychology, big data, and network psychology can be particularly highlighted. At the same time, the relevant research and training in psychology can further penetrate the field of social work, train social workers to master the knowledge and skills of developmental psychology, educational psychology, psychological measurement, psychological counseling, and other related knowledge and skills, improve their professionalism, and provide social psychological services according to the advantages of social work itself. It is suggested that training college counselors, community residents' committees staff, family doctors, people's mediation committee members, and other existing staff should be encouraged, the relevant concept of social psychological services, ethical rules, and practical skills under the unified coordination of the competent unit should be grasped, measures to local conditions to carry out social psychological practice should be adjusted, and the practice of social psychology practice talent reserve can be expanded.

#### 4.2.3. Strengthen the Popularization of Mental Health Education

To strengthen the basic research and scientific popularization of social psychology, the three professional societies can coordinate and form special forces, actively use big data technology and traditional research and measurement technology, and establish a national social mentality database and a national mental health database, to provide data support for the dynamic changes of social mentality and mental health. We can try to construct the social psychological evaluation index such as “China's confidence index” and “national identity index” to comprehensively and accurately measure the effectiveness of community identity construction. At the same time, we should organize professional forces in large and medium campus, enterprises and institutions, urban communities and villages, in various forms of mental health popularization, social mentality, and traditional cultural psychology, inheritance, and innovation activities, let the people in their daily life directly feel professional social psychological services, and improve its subjective happiness, national pride, and cultural self-confidence.

#### 4.2.4. Mobilize All Social Resources

Expand horizontal resources and mobilize social forces to participate in the construction of a social psychological service system. Establish a linkage mode led by governments at all levels and relevant administrative departments, supported by psychological associations and other industries, and participated by social psychological staff in the implementation, and build a basic and comprehensive social psychological service system with communities at different levels as the practice carrier. Led by the local government, colleges and universities to provide intellectual and talent support, industry society supervision, social institutions to provide support, and the government to promote university and community to establish a unique partnership are the basic development modes of Chinese social psychological services and should focus on scientific and deep evidence-based research, form a professional, multitype, multilevel and sustainable social psychological service system.

## 5. Conclusion

In the context of the new crown epidemic, our country is indeed facing this severe mental health challenge. Under the guidance and requirements of the Healthy China strategy proposed by the 19th National Congress of the Communist Party of my country, our country must pay attention to the mental health of the people and strengthen the popularization of mental health education. Therefore, this article mainly proposes the following suggestions for the current mental health problems facing our country. The first is to clarify the social orientation and strengthen the psychoeducational function of social public services. The second is to vigorously develop relevant psychological research with Chinese characteristics. The third is to increase the popularization of relevant research and education and finally to actively use the resources of all sectors of society to develop mental health transactions in all aspects.

## Figures and Tables

**Figure 1:** Mental health education throughout the education stage.

**Figure 2:** Mental health education throughout the whole education stage.

**Figure 3:** The Healthy China action plan.

**Figure 4:** The Healthy China action plan.

**Figure 5:** Schematic diagram of the large health ecosystem.

**Figure 6:** Ten years of mental health changes between oneself and the people around you.

**Figure 7:** Analysis of mental health at different ages.

**Table 1:** Correlations between mental health factors and healthy living.

	Moral cultivation 4.07 (0.59)	Healthy behavior 4.42 (0.43)	No signs of disease 3.76 (0.66)	Adapt and enjoy	
				3.98 (0.58)	*M* (SD)
Health responsibility	0.27^*∗∗*^	0.10	0.34^*∗∗*^	0.28^*∗∗*^	2.38 (0.61)
Self-actualization	0.40^*∗∗*^	0.36^*∗∗*^	0.40^*∗∗*^	0.39^*∗∗*^	2.96 (0.55)
Interpersonal relationship	0.34^*∗∗*^	0.32^*∗∗*^	0.38^*∗∗*^	0.34^*∗∗*^	2.87 (0.49)
Stress coping	0.34^*∗∗*^	0.33^*∗∗*^	0.39^*∗∗*^	0.38^*∗∗*^	2.88 (0.54)
Nutrition	0.32^*∗∗*^	0.27^*∗∗*^	0.40^*∗∗*^	0.31^*∗∗*^	2.71 (0.56)
Sports	0.2^*∗∗*^	0.22^*∗∗*^	0.40^*∗∗*^	0.31^*∗∗*^	2.67 (0.70)
Health promotion lifestyle total score	0.37^*∗∗*^	0.29^*∗∗*^	0.44^*∗∗*^	0.38^*∗∗*^	2.74 (0.51)

**Table 2:** Public trust in different information channels (1∼5 score).

Information channel	Official, media	Large websites	Social, platform	Relatives and friends
Degree of trust	4.34	3.48	3.12	2.83

## Data Availability

The labeled dataset used to support the findings of this study is available from the corresponding author upon request.
